# Modulation of the *Chlamydia trachomatis *In vitro transcriptome response by the sex hormones estradiol and progesterone

**DOI:** 10.1186/1471-2180-11-150

**Published:** 2011-06-25

**Authors:** Ashkan Amirshahi, Charles Wan, Kenneth Beagley, Joanna Latter, Ian Symonds, Peter Timms

**Affiliations:** 1 Institute of Health and Biomedical Innovation, Queensland University of Technology, Kelvin Grove, Queensland 4059, Australia; 2 Faculty of Health, The University of Newcastle, Callaghan, New South Wales 2308, Australia

## Abstract

**Background:**

*Chlamydia trachomatis *is a major cause of sexually transmitted disease in humans. Previous studies in both humans and animal models of chlamydial genital tract infection have suggested that the hormonal status of the genital tract epithelium at the time of exposure can influence the outcome of the chlamydial infection. We performed a whole genome transcriptional profiling study of *C. trachomatis *infection in ECC-1 cells under progesterone or estradiol treatment.

**Results:**

Both hormone treatments caused a significant shift in the sub-set of genes expressed (25% of the transcriptome altered by more than 2-fold). Overall, estradiol treatment resulted in the down-regulation of 151 genes, including those associated with lipid and nucleotide metabolism. Of particular interest was the up-regulation in estradiol-supplemented cultures of six genes (*omcB*, *trpB*, *cydA*, *cydB*, *pyk *and *yggV*), which suggest a stress response similar to that reported previously in other models of chlamydial persistence. We also observed morphological changes consistent with a persistence response. By comparison, progesterone supplementation resulted in a general up-regulation of an energy utilising response.

**Conclusion:**

Our data shows for the first time, that the treatment of chlamydial host cells with key reproductive hormones such as progesterone and estradiol, results in significantly altered chlamydial gene expression profiles. It is likely that these chlamydial expression patterns are survival responses, evolved by the pathogen to enable it to overcome the host's innate immune response. The induction of chlamydial persistence is probably a key component of this survival response.

## Background

*Chlamydia trachomatis *is an obligate intracellular bacterial pathogen that infects the genital and ocular mucosa of humans causing sexually transmitted disease and trachoma respectively. In 2010 the World Health Organization reported 140 million cases of *C. trachomatis *infections occurred worldwide [1]. In females, *C. trachomatis *is a common cause of cervicitis, urethritis, with sequelea including ectopic pregnancy, pelvic inflammatory disease, tubal factor infertility, proctitis and chronic pelvic pain. In males, *C. trachomatis *infections can lead to urethritis, epididymitis and orchitis and it may also contribute to male infertility by directly damaging the sperm [2]. Since approximately 75% of *C. trachomatis *infections in women are asymptomatic, research efforts are mainly focused on females [1,3].

Studies using animal models of genital tract *Chlamydia *infection suggest that the hormonal status of the genital tract epithelium at the time of exposure may influence the outcome of infection. For example, in the commonly used mouse model involving *C. muridarum *infection, pre-exposed of animals with progesterone is required to achieve infection of 100% of the animals [4,5]. Conversely, guinea pigs are more susceptible to infection following pre-treatment with estradiol [6]. Using a rat model, Kaushic *et al. *[7,8] found that in rats infected at either estrus or diestrus, without progesterone pre-treatment, no chlamydial inclusions were observed in either the uterus or vagina. In an *in vitro *model of infection of HeLa cells with *C. trachomatis*, estradiol pre-exposed of cells enhanced both the adherence of chlamydial elementary bodies to the cells as well as the development of chlamydial inclusions [9]. Oral contraceptive use also increases the risk of contracting chlamydial infections compared to women not using contraception [10]. Collectively, these data show that the outcome of chlamydial infection is determined in part by the hormonal status of the epithelium at the time of exposure.

In many cases, chlamydial diseases are associated with a long term or chronic infectious state. In most cases it is difficult to establish whether chronic or recurrent infections arise through the inability of the host to resolve the initial infection or the occurrence of repeated infections with similar species or genotypes. Despite the unresolved nature of the disease etiology, persistence models of chlamydial infection have been studied to provide insight into the nature of chronic disease. Chlamydial persistence is defined as a long-term association between *Chlamydia *and their host cell in which these organisms remain in a viable but culture-negative state [11,12]. Chlamydial persistence is thought to be due in part to a failure to undergo secondary differentiation from RB to EB. Molecular consequences include a 'blockage' in development involving down-regulation of late gene products in persistent infections [13]. The *in vitro *persistence systems often share altered chlamydial growth characteristics, for example, many studies have described enlarged, and pleomorphic RBs that neither undergo binary fission, nor differentiate back to EBs, but nevertheless continue to replicate their chromosomes. Persistent *in vitro *infections have been induced by penicillin treatment, amino acid starvation, iron deficiency, Interferon-gamma (IFN-γ) exposure, monocyte infection, phage infection and continuous culture [12-14]. However, a persistence phenotype has not previously been reported to occur in response to altered levels of sex hormones.

Previous data have demonstrated that the metabolic characteristics of persistent chlamydiae were not the same as those of actively growing organisms [12,15-17]. The results reported from Gerard *et al. *[18] indicated that during the primary phase of active infection, *C. trachomatis *obtain the energy essential for EB to RB transformation, and also for metabolism, from host cells via ATP/ADP exchange. Through active growth of the RB, the organisms acquire ATP not only from the host, but also via their own glycolytic and pentose phosphate pathways. Gerard *et al. *(2002) determined that throughout the initial phase of monocyte infection, prior to the complete establishment of persistence, *C. trachomatis *cells utilized both ATP/ADP exchange and their own pathways to support metabolic needs, even though the overall metabolic rate in the organisms was relatively low. However, when persistence has been established the only source of ATP appears to be the host [18]. This was supported by the finding that, mRNA for glycolytic and pentose phosphate pathway enzymes were absent or severely reduced, suggesting that these systems were partially, if not completely, shut down through persistence. Therefore, *C. trachomatis *seemed to be merely partial energy parasites on their hosts during active growth, however during persistent infection the organisms appeared to be completely dependent on the host for ATP.

In the current study, we utilised a whole genome microarray to study the changes in chlamydial transcriptional response in *in vitro *cultured *C. trachomatis *exposed to either progesterone or estradiol. We found a potentially counter-balancing effect of the two hormones on the chlamydial response.

## Methods

### Hormone supplementation of *Chlamydia*-infected cells

ECC-1: The ECC-1 is a well-differentiated, steroid responsive human endometrial cell line, which was maintained in phenol red-free 1× Dulbecco's Modified Eagle Medium/Ham's F12 nutrient mix (DMEM/F12 - 1:1) (Invitrogen, Carlsbad, CA, USA).

HEp-2: The HEp-2 cell line is a human epithelial cell line, which was maintained in 1× DMEM containing phenol red, 4.5 g/L D-glucose, 110 mg/L sodium pyruvate, and 584 mg/L L-glutamine, and supplemented with 500 U/ml penicillin G sodium/5,000 μg/ml streptomycin sulphate (Invitrogen).

### Hormone preparation

Lyophilised progesterone and 17β-estradiol (Sigma-Aldrich, St. Louis, MO, USA) were solubilised in absolute ethanol to 1 mg/ml stock. Serum levels of female sex hormones, estradiol and progesterone, fluctuate throughout the menstrual cycle. In this study mean physiological concentrations of 17β-estradiol (200 pg/ml) and progesterone (20 ng/ml), adapted from Williams Textbook of Endocrinology were further diluted using phenol red-free 1× DMEM/F12 medium (Invitrogen), supplemented with 10% charcoal/dextran-treated FBS (Hyclone). Once the ECC-1 cells had reached 100% confluence, average physiological concentrations of 17β-estradiol, progesterone, and a combination of 17β-estradiol and progesterone (1:1) were added to respective flasks. This hormone exposure was continued throughout the duration of chlamydial infection. Although the physiological concentration of progesterone is higher than estradiol, in this study a combination of 1:1, estradiol and progesterone, was chosen as starting point to merely determine the effect of both hormones together. Cells were then incubated for 24 hrs before continuance of experiments.

### *C. trachomatis *serovar D growth and propagation

*C. trachomatis *serovar D was grown, maintained and further propagated to create *C. trachomatis *serovar D stock. *C. trachomatis *was semi-purified from the infected HEp-2 cells via sonication and vortexing. ECC-1 cells were used for *C. trachomatis *serovar D titration. Infected cells were stained utilising the CelLabs Chlamydia Cel LPS staining kit, containing the fluorescein isothiocyanate (FITC)-labelled mouse monoclonal antibody specific for chlamydial lipopolysaccahride (LPS) (CelLabs, Brookvale, Australia), according to manufacturer's instructions.

### RNA Extraction

Total RNA was extracted 48 hrs post infection from infected ECC-1 cells using the Trizol^® ^reagent protocol (Invitrogen) and then treated with DNase. Eukaryotic RNA was removed from total RNA using the Dynabead (poly A^+ ^purification kit) (Dynal Biotech ASA, Oslo, Norway) according to manufacturer's instructions and the bacterial mRNA re-suspended in DEPC water. Approximately 2 μl of the bacterial mRNA solution was removed to determine the quality and quantity of RNA, using a NanoDrop^® ^Spectrophotometer (NanoDrop Technologies^®^, Wilmington, DE, USA) and associated NanoDrop ND-1000 3.2.1 software (Coleman Technologies Inc., Glen Mills, PA, USA). Extracted RNA was determined to be of high purity, as indicated by the absorbance ratio (A260:A280) being very close to 2.00. The quantity of RNA extracted indicated amplification was not required prior to microarray analysis as the concentration of RNA was sufficient for our experiments.

### Whole transcriptome analysis by Affymetrix microarray

The bacterial mRNA was sent to the AGRF (Australian Genome Research Facility, Melbourne, Australia) for microarray analysis. *In vitro *RNA transcription was performed to incorporate biotin-labelled ribonucleotides into the cRNA transcripts using the ENZO RNA transcript labelling kit. Labeled cRNAs were purified using the Qiagen kit (according to manufacturer's instructions) and then fragmented to approximately 50 to 200 bp by heating at 94°C for 35 min. Fifteen micrograms (15 μg) was then hybridized to a *Chlamydia *whole genome Affymetrix Custom array. The array is an Affymetrix oligonucleotide array format of 1800 features, covering the full *C. trachomatis *genome (875 genes) and containing 8-11 oligonucleotides per target gene, each designed for optimal hybridization to *C. trachomatis *and/or *C. pneumoniae *and screened for non-specific hybridization against the full human and mouse genomes. After hybridization and subsequent washing using the Affymetrix Fluidics station 400, the bound cRNAs were stained with streptavidin phycoerythrin, and the signal amplified with a fluorescent-tagged antibody to streptavidin (Performed by AGRF). Fluorescence was measured using the Affymetrix scanner and the results analysed using GeneChip 1.4 analysis software, resulting in the detection of 1175 genes. A total of 16 chlamydial arrays were analysed with the 4 culture conditions (no hormone, E, P, E+P) × four replicates. The entire microarray data recorded in Gene Expression Omnibus (GEO) database with accession number GSE24119.

### Quantitative RT-PCR

Quantitative Real-Time PCR was used to validate the microarray data for 20 selected target genes. Each primer pair was used to generate amplicon standards by amplifying previously generated *C. trachomatis *cDNA. cDNA generation was performed using the SuperScript^® ^III Reverse Transcriptase technique (Invitrogen, Carlsbad, CA, USA). One μg of template was added to the PCR mixture containing 0.15 μM of gene specific forward and reverse primers, 1 × SYBR Green reaction mastermix, before being made up to a final volume of 25 μL with distilled water. The mix is optimized for SYBR Green reactions and contains SYBR Green I dye, AmpliTaq DNA Polymerase, dNTPs and optimized buffer components. Cycling parameters for all reactions were as follows: denaturation at 95°C for 10 min; 40 cycles of denaturation at 95°C for 15 sec and 1 min of annealing and extension at 60°C; and melting curve analysis from 60°C to 95°C. The Rotor-Gene 6000 fast real-time PCR system (Corbett) was used for relative quantification of cDNA copies for the 20 selected genes and an internal reference gene (16S rRNA) was used in all experiments. Quantitation was carried out by using a standard curve based on serial dilutions of the amplicon standards covering 6 logs. Real-time PCR templates for each gene of interest included fresh dilutions of the amplicon standards, 8 cDNA samples (2 × 4 samples per experiment) and distilled water as a negative control. All reactions were performed in triplicate. Reaction tube mastermixes were prepared as per the preparation of amplicon standards described above.

Each gene array profile indicated the expression level of each gene under the differing experimental conditions. To identify genes with similar expression profiles mathematical clustering methods were used, with the resulting hierarchy displayed as dendrograms. 16s rRNA was used as an internal control. The use of an internal control was necessary as the number of genes expressed under different hormonal conditions varied substantially and no single gene was constitutively expressed. This method of normalization was particularly important in comparing samples grown in charcoal-stripped, hormone-free media to those in hormone-supplemented cultures.

#### Microarray data accession number

The entire microarray data recorded in Gene Expression Omnibus (GEO) database with accession number: GSE24119.

## Results and discussion

### Whole transcriptome microarray data confirmed by qRT-PCR analyses

We used a whole genome Affymetrix microarray approach to measure the transcriptional responses of *C. trachomatis *grown in ECC-1 cells supplemented with the female sex hormones, estradiol and progesterone. The resultant data was extracted and filtered through Affymetrix's Gene Chip Operating System (GOCS) version 1.4, and processed using the MAS5 algorithm. Candidate lists of genes were further refined by selecting genes with a greater than 2-fold up/down-regulation and a *p*-value of <0.05. Replicate data sets were processed individually and then cross-correlated with each other to find statistically significant changes in gene expression. A total of 16 chlamydial arrays were analysed, with the four culture conditions (no hormone, E, P, E+P), enabling us to have four replicates for each test condition. To confirm the accuracy and reliability of our microarray data, we chose 19 genes that were either up or down-regulated by microarray for analysis by quantitative RT-PCR (Table 1). For 17 of these 19 genes there was complete agreement between the microarray results and the qRT-PCR results. In all cases the fold changes measured by qRT-PCR were larger than those recorded using the microarray assay. For the two genes that were not consistent between the two methodologies, the microarray method gave a down-regulation of transcription whereas the qRT-PCR method showed no change in the transcriptional response.

**Table 1:** Comparison of expression folds change obtained by microarray analysis with fold change obtained by qRT-PCR.

Gene name	Affymetrix fold change	qRT-PCR fold change
*gseA*	13.30 up	27.94 up
*nqr2*	9.20 up	17.32 up
*ytgD*	9.05 up	14.07 up
*ydaO*	5.98 up	12.51 up
*pdhA*	5.78 up	17.30 up
*recA*	4.12 up	7.92 up
*lplA 2*	3.89 up	7.41 up
*trpB*	3.80 up	11.87 up
*incA*	3.10 up	18.04 up
*fli1*	2.25 up	6.80 up
*sdhB*	22.53 Down	6.8 Down
*trxB*	31.44 Down	5.19 Down
*pyrH*	21.54 Down	No change
*miaA*	33.91 Down	11.74 Down
*cysS*	19.09 Down	7.03 Down
*nrdA*	30.06 Down	5.16 Down
*pbp3*	33.53 Down	9.43 Down
*ychF*	21.29 Down	No change
*yggV*	31.84 Down	12.11 Down

### Approximately 25% of the *C. trachomatis *transcriptome is altered in response to estradiol or progesterone exposure *in vitro*

A significant percentage (approximately 25%) of the *C. trachomatis *transcriptome was altered in response to both hormones. Using a 2-fold change as a cut-off, 63 genes (7%) were up-regulated in response to estradiol while 151 genes (17%) were down-regulated (Table 2). A similar percentage (but different subset) of the transcriptome was altered under progesterone exposure, with 85 genes (10%) being up-regulated and 135 genes (15%) being down-regulated. This represents around 25% of the transcriptome as a whole, being altered by either hormone alone. When the cut-off was set at 3-fold, 18-20% of the transcriptome was still changed in response to the sex hormones, but this level dropped to 12% when a 5-fold cut-off is used. The full microarray dataset is provided in the GEO database.

**Table 2:** Summary of *Chlamydia trachomatis *up-regulated and down-regulated genes in response to estradiol or progesterone exposure.

	Estradiol	Progesterone
	
	No. of genes/% of genome	No. of genes/% of genome
**Up regulated**		
A: > 2-fold, change	63 (7%)	85 (10%)
B: > 3-fold change	52 (6%)	77 (9%)
C: > 5-fold change	22 (2.5%)	49 (5.5%)

**Down regulated**		
A: > 2-fold, change	151 (17%)	135 (15%)
B: > 3-fold change	138 (15.7%)	117 (13%)
C: > 5-fold change	98 (11%)	81 (9%)

(A) 2-fold cut-off, (B) 3-fold cut-off, (C) 5-fold cut-off.

### Estradiol exposure results in the specific down-regulation of lipid and nucleotide metabolism pathways

In the estradiol-exposed cultures, 151 genes were down-regulated more than 2-fold, while 63 genes were up-regulated more than 2-fold during the same period. Of these 213 altered genes, more than 52% were hypothetical proteins, with no known homologues outside the chlamydiae. Even though nearly 30% of the chlamydial genome is composed of hypothetical genes, the fact that 52% of these genes altered their expression by more than 2-fold in response to estradiol exposure suggests that many of the key changes are uniquely associated with *Chlamydia*. The five top up-regulated genes (ie. showing the largest fold change) included the Nqr2 subunit of Na-translocating NADH-quinone reductase complex (*nqr2*) [9.26 fold], UDP-N-acetylmuramoylalanine-D-glutamate ligase, putative (*murC/ddlA*) [9.31 fold], V-type ATPase, subunit D, putative (*atpD*) [10.23 fold], arginine transport system substrate-binding protein (*artJ*) [10.96 fold], and putative glycerol-3-phosphate acyltransferase (*plsX*) [16.53 fold]. In addition, the five genes that showed the largest down-regulation of mRNA expression profile include cell division protein FtsI (*pbp3*) [35.54 fold], nucleoside-triphosphatase (*yggV*) [31.84 fold], ribonucleoside-diphosphate reductase alpha chain (*nrdA*) [30.06 fold], GTP-dependent nucleic acid-binding protein (*ychF*) [21.29 fold], and succinate dehydrogenase iron-sulfur subunit (*sdhB*) [18.82 fold].

When the up- and down-regulated genes were input into the KEGG Pathway database http://www.genome.jp/kegg/pathway.html, using the known or predicted chlamydial pathway information, some clustering of transcriptional responses was evident (Table 3). Estradiol clearly induced an overall down-regulation of chlamydial fatty acid biosynthesis, with seven genes being down-regulated at least 2-fold (*accB*, *fabF*, *lipA*, *fabG*, *lplA_2*). Estradiol also resulted in a marked down-regulation of the genes involved in chlamydial nucleotide (purine and pyrimidine) metabolism (*adk*, *dnaE*, *dut*, *nrdA*, *surE*, *yggV*, *rpoC*, *ygfA*, *dut*). In addition, we also observed a more minor down-regulation in cofactor and vitamin metabolism pathways (*hemC*, *hemN*-*1*, *yggV *and *folD*).

**Table 3:** Categorisation of the up- and down-regulated genes into pathways, as per KEGG.

	Total	Up-regulated		Down-regulated	
		
		Estradiol	Progesterone	Estradiol	Progesterone
Energy metabolism	14	3	4	6	4
Carbohydrate metabolism	23	2	9	1	-
Lipid metabolism	27	1	2	7	8
Nucleotide metabolism	29	-	1	16	3
Amino acid metabolism	30	3	8	3	3
Metabolism of other amino acids	4	-	-	-	-
Metabolism of cofactors and vitamins	33	-	1	6	3
Glycan biosynthesis and metabolism	16	2	6	1	2
Biosynthesis of secondary metabolism	15	1	1	3	4
		**12**	**32**	**43**	**27**

The numbers represent the number of pathways (not genes) affected following exposure with either Estradiol or progesterone.

Taken together, this overall down-regulation of key pathways is suggestive of a persistence phenotype. The normal chlamydial developmental cycle can be altered under stressful conditions, leading to the formation of aberrant bodies (ABs) which are inhibited in their differentiation back to infectious EBs [11]. Molecular consequences include a 'blockage' in development involving down-regulation of late gene products in persistent infections [19].

The *omcB *and *trpB *genes are currently the most reliable general markers of chlamydial persistence [12-14,20-22]. The down-regulation trends reported in this project, for these genes under estradiol supplement, were consistent with previous data in the microarray study of IFN-γ-mediated *C. trachomatis *serovar D persistence [13]. It has previously been shown that *trpA *and *trpB *are two genes known to be involved in chlamydial persistence [12,20]. Hogan *et al. *[12] showed that the expression patterns of these two genes were mostly up-regulated in chlamydial persistence. While the expression level of *trpB *in our experiment indicated a similar up-regulation, the expression levels of *trpA *did not change. As an additional strategy, we attempted to identify chlamydial genes involved in ADP/ATP exchange and energy source pathway reactions in the *C. trachomatis *genome. This analysis revealed six targets which may be involved in chlamydial persistence (a) two genes encoding proteins involved in the glycolysis pathway (*pyk*, *yggV*) (b), two genes (*cydA*, *cydB*) encoding proteins involved in the electron transport system, and (c) two genes encoding proteins involved in the production of tryptophan synthase subunits. Previous data have demonstrated that the metabolic characteristics of persistent chlamydiae were not the same as those of actively growing organisms [12,15-17]. The results reported from Gerard *et al. *[18] indicated that during the primary phase of active infection, *C. trachomatis *obtains the energy essential for EB to RB transformation, and also for metabolism, from host cells via ATP/ADP exchange. Through active growth of the RB, the organisms acquire ATP not only from the host, but also via their own glycolytic and pentose phosphate pathways. Gerard *et al. *(2002) showed that throughout the initial phase of monocyte infection, prior to the complete establishment of persistence, *C. trachomatis *cells utilized both ATP/ADP exchange and their own pathways to support metabolic needs, even though the overall metabolic rate in the organisms was relatively low. However, when persistence has been established, the only source of ATP seemed to be the host [18]. That is, mRNA for glycolytic and pentose phosphate pathway enzymes were absent or severely reduced, suggesting that these systems were partially, if not completely, shut down during persistence. Therefore, *C. trachomatis *seems to be only partial energy parasites on their hosts during active growth, however during persistent infection, the organisms appear to be completely dependent on the host for ATP.

Most notably in our current project, *pyk *and *yggV *were strongly down-regulated (3-fold and 10-fold respectively) following supplementation with estradiol, which may contribute to a reduction in the rate of glycolysis biosynthesis during persistence. Two other well known chlamydial persistence genes (*cydA*, *cydB*), which play a part in the electron transport system were also down-regulated (8-fold and 4-fold respectively) in the presence of estradiol.

The other key persistence-suggestive change was observed at the morphological level. It has been previously reported by several authors [13,23,24] that chlamydiae show abnormal morphology under persistence conditions. We analysed both un-exposed as well as hormone-exposed *C. trachomatis *infected ECC-1 cell cultures using Transmission Electron Microscope (TEM) analysis (Figure 1). Under normal cell culture conditions (ie cell culture media supplemented with FCS) we observed normal chlamydial inclusion growth and development as depicted by a mixture of characteristic RBs and EBs of normal size and shape (Figure 1, Panel A). By comparison, when we grew the chlamydiae in charcoal stripped foetal calf serum (hormone free media), supplemented with estradiol, we observed typical chlamydial persistence inclusions containing aberrant, enlarged RBs which had not differentiated into EBs (Figure 1, Panel C). The morphological features that we observed associated with hormone-mediated persistence demonstrate similarities to those observed by others for persistence induced by IFN-γ and penicillin.

**Figure 1:** **Transmission electron micrographs of *C. trachomatis *inclusion development in ECC-1 cells at 48 hours under different hormonal conditions estradiol and/or progesterone**. (A) ECC-1 cells grown in normal FCS supplemented cell culture. Typical RB forms are present at 24 hours post infection (B) No hormone supplemented stripped FCS media. Once again normal RB morphology was observed under this condition; RBs appeared similar to normal FCS supplemented cell culture. (C) Estradiol supplemented, RBs were distinctly different, appearing as large aberrant form. Estradiol supplementation of infected cells, resulting in smaller inclusions containing enlarged, atypical RB forms (arrows). (D) Progesterone supplemented, shape and morphology of RBs were normal including binary fission. Morphological examination of progesterone exposed cultures with TEM did not show any evidence of aberrant, persistent forms. Magnification: × 20K, marker represent 200 nm.

### Progesterone exposure induces an up-regulated energy utilising chlamydial response

Overall, 85 chlamydial genes were observed to have two-fold or greater up-regulated gene expression levels in the presence of progesterone. The five top genes that were observed with this mRNA expression profile encode for proton or sodium-glutamate symport protein (*gltT*) [33.4 fold], the putative glycerol-3-phosphate acyltransferase (*plsX*) [16.17 fold], glucose inhibited division protein (*lplA_2*) [11.9 fold], NADH-quinone reductase complex (*nqr2*) [10.95 fold] and polynucleotide adenylyltransferase (*pcnB_1*) [10.75 fold]. In addition to these 85 genes, 135 chlamydial genes were observed to have a reduced gene expression profile in response to the presence of progesterone. The five top down regulated genes include exoribonuclease II (*vacB*) [67.96 fold], isopentenylpyrophosphate transferase (*miaA*) [33.91 fold], cysteinyl-tRNA synthetase (*cysS*) [33.64 fold], thioredoxin reductase (*trxB*) [33.44fold], and ribonucleotide-diphosphate reductase subunit alpha (*nrdA*) [29.25 fold]. 103 genes had unknown annotated functions (hypothetical genes).

By comparison to the estradiol response, which resulted in a down-regulation of fatty acid and nucleotide metabolism pathways, progesterone exposure had no or little effect on these pathways but did result in a significant up-regulation of the TCA cycle and glycolysis pathways (Table 3). In some aspects the progesterone response was opposite or counter-balancing to the estradiol response. Progesterone resulted in a general up-regulation of carbohydrate metabolism pathways as well as an up-regulation of amino acid metabolism pathways.

The progesterone-mediated response mounted by *Chlamydia *reflects the host's flux of metabolites. Progesterone has been reported to have a suppressive effect in general on estradiol [25], and after prolonged exposure, it appears that *Chlamydia *is diverting specific pathways to compensate. From the top five up-regulated genes, three genes are associated with *Chlamydia*-specific salvage pathways: *lplA_2 *for regeneration of lipoic acid; and *plsX *for the formation of glycerophospolipids and phosphotidylcholine regeneration; *nqr2 *for the regeneration of NAD(P)H and free-radicals. The association with the top five down-regulated genes appears to align with control at the transcriptional/translational level. For example, the gene encoding *miaA *and *cysS *have associated functions with translation, through transfer RNA molecules. *nrdA *plays an important role in nucleotide regeneration and our observation that expression of this gene was down 29-fold, suggests that one mechanism being employed by *C. trachomatis *is to reduce cellular multiplication.

While these chlamydial transcriptome changes might be a direct result of the effect of the hormones on the chlamydiae it is likely that the major effects are indirect, via the host cells. As an intracellular pathogen, most of the chlamydial response to the hormones is most likely an indirect response to changes in the host cells. In a parallel study (Wan *et al.*, manuscript submitted) we have analysed the host cell response to these hormones and have found a cascade of changes. It is likely therefore that the chlamydial transcriptome changes are in response to these host cell changes. It is known that hormones have a major effect on host cell innate immune pathways. For example, the expression of antimicrobial peptides such as human defensin 5 (HD-5 [26]), lactoferrin [27,28], and secretory leukocyte protease inhibitor (SLPI) [29] are all influenced by changes in female sex hormones, as is the recruitment of neutrophils, macrophages and NK cells into the reproductive tract [30]. Furthermore, chlamydial infection of progesterone-exposed endocervical cells results in increased mRNA levels for multiple chemokines, cytokines as well as up-regulation of various interferon pathways in these cells (Wan *et al. *manuscript submitted) suggesting that the chlamydial changes may be in response to the altered host cell environment. In the present study we analysed the effects of either progesterone or estradiol separately. In reality, both hormones are continually present, but their levels fluctuate during the various stages of the estrous cycle. This hormonal cycling may have the effect of causing the chlamydiae to alternate between cycles of productive growth and cycles of persistence or dormancy. Given the 28 day duration of the human female menstrual cycle and the 2-3 day growth cycle of *C. trachomatis*, such cycling is a real possibility and may be of survival benefit to the chlamydiae.

## Conclusions

This is the first study to demonstrate transcriptional analysis of *Chlamydia trachomatis *genes under different hormonal conditions. Previous studies provided evidence that the hormonal environment at the time of pathogen exposure can have anclinical effect on the outcome of a microbial infection in the genital tract. In the current experiments, we examined the effect of the hormonal environment on (a) *C. trachomatis *gene expression and (b) the type of inclusions that develop. In our experiments, evidence of long-term persistent chlamydial infections was observed. Collectively our data suggest that hormonal supplementation; estradiol in particular, may directly or indirectly play an important role in the development of chlamydial persistence. The data may help to explain why infections are more common in the estrogen-dominant phase of the menstrual cycle and suggest that estradiol favours the development of persistent infections that may allow *Chlamydia *to; (a) resist common antibiotic therapy and (b) survive the innate immune response to infection, thereby facilitating repeated reactivation of infection that drives damaging immunopathology.

## Competing interests

The authors declare that they have no competing interests.

## Authors' contributions

AA carried out the molecular genetic and microarray studies, participated in the microarray analysis and drafted the manuscript. CW designed microarray chip and participated in the microarray analysis. KB conceived the study and revised the manuscript critically for important intellectual content. JL participated in the cell culture and provided the initial samples. IS revised the manuscript critically for important intellectual content. PT participated in the design of the study, project coordination and helped to draft the manuscript. All authors read and approved the final manuscript.
